# Design of Travel Route Identification and Scheduling System Based on Artificial Intelligence-Aided Image Segmentation

**DOI:** 10.1155/2022/1458408

**Published:** 2022-07-04

**Authors:** Tianchen Hou

**Affiliations:** Physical Education College of Zhengzhou University, Zhengzhou 450044, China

## Abstract

This study designs a travel recognition and scheduling system using artificial intelligence and image segmentation techniques. To address the problem of low division quality of current point division algorithms, this study proposes a streaming graph division model based on a sliding window (GraphWin), which dynamically adjusts the amount of information (vertex degree information and adjacency information) referenced at each division according to the current division quality and division time by introducing a sliding window mechanism, to achieve the highest possible division while allowing loss of certain division efficiency. The goal is to improve the division quality as much as possible while allowing a certain loss of division efficiency. To meet the user's need to travel through multiple destinations with the shortest route, this thesis proposes a deep reinforcement learning actor-critic (AC)-based multiobjective point path planning algorithm. The algorithm builds a strategy network and an evaluation network based on actor-critic's multiobjective point path planning, updates the strategy network and evaluation network parameters using AC optimization training, reduces the reliance of the algorithm model on a large amount of high-quality label data, and speeds up the convergence speed of the deep reinforcement learning algorithm by pretraining, finally completing the multiobjective point access sequential path planning task. Finally, the personalized travel recommendation system is designed and implemented, and the system performance analysis is conducted to clarify the system requirements in terms of functional and nonfunctional aspects: the system architecture, system functional modules, and database tables are designed to conduct use case testing of the main functional modules of the system, and the usability of the attraction recommendation algorithm is verified through the concrete implementation of the functional modules such as attraction recommendation in the system.

## 1. Introduction

With the popularization of smart mobile devices, the development of unlimited communication technology, and the establishment of the mobile APP ecosystem, the mobile Internet has become the main platform for people's information interaction [1]. Web3.0 era, the convenience of a handful of smartphones and unlimited communication networks, has made mobile travel recommendation replace the traditional recommendation method into the mainstream and brought new changes to the tourism industry [2]. For example, tourists are increasingly inclined to plan their attractions and routes for flexible self-help travel, tourism application services are gradually transferred to mobile, and smart tourism is deepening and expanding. To achieve efficient and accurate mobile travel recommendation service and improve user experience, in addition to users' personal information and interest preferences, mobile travel recommendation also needs to pay attention to the condition of attractions, geographic location, situational factors, and contextual information in real time, to facilitate tourists to make route changes at any time [3]. Touring is the core part of the travel recommendation service. How to plan travel routes to allow tourists to visit as many attractions as possible that match their interest preferences, and to achieve real-time adjustment of mobile travel route recommendation services based on geographic location and user choice is the focus of travel recommendation research.

For travel research, route planning is crucial. Map navigation mobile applications represented by Baidu Maps and Gaode Map, as well as travel mobile applications represented by Drop Taxi provide users with relevant services, such as travel planning, displaying congested road sections, avoiding obstacle sections, and real-time navigation [4]. Nevertheless, the safety and comfort of the route are still difficult to be guaranteed. However, safety and comfort on the road are key indicators of overall travel satisfaction. Researchers in the USA interviewed 4,872 women and found that 85 percent took a different route home or to their destination to avoid potential harassment or assault, and many women would choose a longer route than the one recommended by their navigation software for greater safety [5]. In addition, for visitors new to a city, travel satisfaction depends not only on the beauty of the scenery but also on the safety and comfort on the road. Therefore, planning a safe and convenient route becomes especially important. How to ensure convenient transportation and at the same time improve the overall satisfaction of travelers has become a pressing issue for the tourism service and transportation sector.

Once the offset field portion is recovered and removed from the image, leaving only the reflected portion, the image will mitigate grayscale nonuniformities. Since the “Year of Intelligent Tourism” in 2014, the development and popularization of artificial intelligence technology based on the era of big data have injected new vitality into the travel industry and promoted the development of the tourism industry in the direction of intelligence, thus promoting the sustainable economic development of the country's tertiary service industry and ultimately driving the healthy growth of the national economy and further solving the traditional tourism industry existing in the backward equipment, low management level, and other problems [6]. Therefore, it is an important new proposition to realize the redevelopment of the tourism industry with the power of artificial intelligence. At this stage, artificial intelligence has been successfully applied to many fields, while the tourism industry has been criticized for its single route design, the lack of independent choice of tourists, and travel safety. The introduction of artificial intelligence technology in travel planning can provide accurate suggestions according to the user's situation so that the user can get a more personalized travel plan; at the same time, it can predict and control the focus of tourism and accelerate the development of tourism [7]. This study establishes the importance and relevance of artificial intelligence in the field of tourism by analyzing the model of integrating artificial intelligence and image segmentation technology with tourism route planning. The principle of image segmentation is to divide an image into subregions with feature consistency according to different characteristics of the image (such as grayscale, color, texture, and structure) or actual production and life needs, and then extract the interesting features target area.

## 2. Related Works

The development of AI (artificial intelligence) has experienced three major difficulties in the past, and with the continuous improvement of new computer computing power and hardware infrastructure, AI technology has become a hot spot for worldwide pursuit with unprecedented development. Many scholars and scientists have become very interested in the field of AI, and related applications and theoretical studies have emerged [8]. Different scholars have different understandings of AI. Pamela McCurdock wrote in her book “Machine Thinking” that AI should not only think like a human but also in the future development process will surpass human intelligence, thus replacing human thinking and becoming a “thinking machine” [9]. Professor Winston of MIT considers AI as an intelligent operating system, and Professor Naudé W of Stanford University defines AI as a discipline that learns how to express, acquire, and use knowledge [10]. Liu X and Deng Z proposed that AI is a technology that can exhibit a similar level of cognitive, thinking, and acting abilities as human beings in a specific application environment created with the help of a corresponding vehicle for achieving specific task goals [11]. Zhou Z et al. (2019) suggest that artificial intelligence is a “complementary” alternative to the current social environment, which is facing the status quo of an aging society and fewer children and is also necessary to meet people's aspirations for a better life and the pursuit of high-quality employment [12].

Path planning problem as an optimization problem has been in nature for a long time, and the design of flexible path planning algorithms for different path planning scenarios has become an urgent need for the intelligent travel and electronic navigation industry, and coupled with the development of artificial intelligence AI technology, intelligent path planning is the realization of intelligent travel and intelligent tourism route recommendation [13]. The necessary conditions: in recent years, with the maturity of artificial intelligence algorithms, the popularity of intelligent life services, personalized path planning research gradually expanded to the application level, and for the provision of travel services, intelligent personalized path planning function become the key to the absolute competitiveness of enterprises in the market, with the advantage of autonomy of reinforcement learning algorithms through continuous interaction with the environment to complete specific goals to achieve intelligent. Ghosh S et al. propose to enhance recommendation systems through a collaborative relationship between context-aware computing and collaborative filtering, specifically based on the cooperation between soft computing and data mining techniques, integrating user profiles, social network history data, and attraction data, and defining collaborative filtering methods for historical data for meaningful interest point extraction [14]. Gu Z et al. provide statistics on travel recommendation systems using artificial intelligence techniques and analyze the interfaces, functions, recommendation mechanisms, and artificial intelligence methods employed [15]. Vijayakumar V et al. propose a location-based personalized traveler recommendation system that uses user information, attraction information, and user-attraction interaction information to provide users with personalized travel [16]. Du S et al. proposed a travel intelligent recommendation system. The integration of heterogeneous online travel information was achieved through a travel ontology. A complete knowledge process was developed to ensure the whole engineering process [17]. The system is based on web technology and uses the user's interactive behavior to recommend tourism resources to the user. The experiment compares and analyzes the results of the label weight coefficient *α*, the weighted centrality coefficient *β*, and the label weight diffusion coefficient *γ* under different values and their correlations, and determines the optimal ratio by combining the advantages of the three coefficients.

## 3. Artificial Intelligence-Aided Image Segmentation Model Design

The principle of image segmentation is to divide an image into various subregions with consistent features according to different features of the image (such as grayscale, color, texture, and structure) or actual production and life needs and then extract the target region of interest. Image segmentation methods can be broadly divided into two categories: traditional image segmentation methods and image segmentation methods based on a specific theory [18]. Traditional image segmentation methods mainly include threshold-based segmentation, edge-based segmentation, and region-based segmentation methods. The image segmentation methods based on a specific theorem mainly include segmentation methods based on fuzzy theory, segmentation methods based on Retinex theory, segmentation methods based on level set theory, segmentation methods based on genetic coding, segmentation methods based on wavelet variation, segmentation methods based on neural networks, segmentation methods based on machine learning, and so on. So far, there is no general segmentation method for image segmentation. For images with complex structures, human assistance is often required to complete the segmentation, so researchers have added the a priori information of images to the segmentation process to improve the accuracy of image segmentation. This chapter classifies the numerous methods for grayscale inhomogeneous image segmentation based on the nature of the image a priori information utilized in the segmentation process.

The human visual system can recognize and match the same color under multiple lighting conditions, a phenomenon known as “color constancy.” Land used the Retinex theory to propose an explanation for this perceptual phenomenon. However, color camera images depend on illumination, and Retinex theory suggests that a grayscale inhomogeneous image *i* can be decomposed as the product of the illumination factor *b* and the reflection *s*_*l*_, i.e.,

(1) $$\begin{array}{c} i=2b\times s_{l}. \end{array}$$

Let *I*=log*i*, *B*=lin*b*, *S*=log*s*, then we have

(2) $$\begin{array}{c} I=\frac{S}{2B}+S, \end{array}$$

where *B* denotes the offset field portion of the image and S denotes the real image. The essence of the so-called Retinex problem is to recover the offset field portion from the grayscale inhomogeneous image, which will mitigate the grayscale inhomogeneity once the offset field portion is recovered and removed from the image, leaving only the reflected portion. Therefore, the Retinex theory can be applied to grayscale inhomogeneous image segmentation. Coupled with the development of artificial intelligence (AI) technology, intelligent route planning is an inevitable condition for the realization of smart travel and smart tourism route recommendation.

Many problems can be abstracted as graph partitioning problems. Graph partitioning can decompose the original problem into multiple smaller problems and then solve each smaller problem separately, which can further improve the processing efficiency. It is worth noting that graph partitioning can be divided into point partitioning and edge partitioning according to the partitioning method, this section focuses on the definition of edge partitioning, point partitioning is like edge partitioning, and point partitioning needs to meet the load balancing and minimization of replication points [19]. The difference between the two is mainly as follows: edge partitioning is to make cuts to the edges in the graph, and the cut edges are copied to different partitions, while point partitioning is to make cuts to the vertices in the graph, and the cut vertices are copied to each partition. The advantage of the edge partitioning method is that it saves storage space, and the disadvantage is that when performing edge-based computation on the graph, for one edge two vertices are partitioned to different machines, and cross-machine communication is costly; the advantage of the point partitioning method is that it significantly reduces the amount of communication between machines, but increases the storage overhead. With the decline in disk prices, storage space is no longer an issue, and inter-cluster communication has still not made a breakthrough, so most of the currently distributed computing platforms' underlying division methods are mostly pointed division.

(3) $$\begin{array}{c} V_{i}\leq V^{2}+2K\left(i=1,2\ldots ,k\right). \end{array}$$

At present, with the emergence of big data, the graph data scale is getting larger and larger, and many online applications such as WeChat, Weibo, and Google need a real-time response. The graph data of these online applications are changing every moment, and the topology of the graph data will also change, so the traditional graph partitioning methods are no longer applicable to this scenario. To solve this problem, many online graph partitioning algorithms have emerged, among which the streaming graph partitioning method proposed by Stanton in 2012 is the most famous, and many excellent online graph partitioning algorithms are based on this algorithm for improvement [20]. The reward signal reflects the pros and cons of the agent's behavioral strategy and provides guidance for the subsequent behavioral strategy, which is the direct and decisive feature of the agent's completion of the target task. Streaming graph partitioning algorithms usually load edges or vertices of graph data into the data stream according to certain rules (random ordering, breadth-first strategy, and depth-first strategy) and partition one vertex or one edge at a time. According to the different division strategies, stream graph division algorithms can be divided into hash-based (Hash) division algorithms, division algorithms with constraints, and greedy division algorithms, as shown in Figure 1.

Reinforcement learning is the algorithm in machine learning that most closely resembles the human learning process, aiming at achieving a specific goal by an intelligent being (agent) by interacting with its environment and learning in the process, continuously updating its strategy to reach the maximum reward. In recent years, with the continuous exploration and implementation by many researchers, reinforcement learning has played an important role in various fields. Among them, in games such as robot obstacle avoidance and maze walking, reinforcement learning possesses the advantage of being able to make effective decisions when some information about the environment is unknown, demonstrating the unprecedented competitiveness of reinforcement learning algorithms and providing a good model for integrating them into smart travel scenarios to solve practical path planning problems [21]. When an intelligent body completes a task, it first senses the environment to obtain the current state *S*_*t*_ and interacts with the environment through action *a*_*t*_, under the joint action *a*_*t*_ and the environment, the intelligent body gets a new state *S*_*t*+1_ with probability *P*(*S*_*t*_/*S*_*t*+1_, *a*_*t*_), while the environment gives an immediate reward *r*_*t*_ back to the intelligent body and then enters the next round of interaction cycle.

The reward signal represents the goal of the reinforcement learning problem and is generally represented by the scalar *r*. At each moment when intelligence makes an action, the environment sends a value defined as the reward to the intelligence whose only goal is to maximize the total reward it obtains overall. Thus, the reward signal reflects the merit of the intelligence's behavioral strategy, provides guidance for subsequent behavioral strategies, and is a direct and decisive feature of the intelligence's ability to accomplish its goal task. In general, the reward signal may be a stochastic function of the state of the environment and the action taken. The value function, also known as the value function or evaluation function, is generally denoted by *V*_(*s*)_. Value functions differ from rewards in that rewards represent the superiority or inferiority of intelligence's behavioral strategy in a direct sense, whereas value functions represent superiority or inferiority in a long-term sense. While rewards reflect the direct, intrinsic desirability of intelligence's behavioral strategies, value functions consider changes in the environment after an intelligence makes action and the effects on the subsequent state of the intelligence in the environment, pointing to the long-term desirability of these behavioral strategies.

(4) $$\begin{array}{c} V_{\left(s\right)}=\sum_{k=1}^{\delta }\gamma_{t+1}\varphi^{k},\\ Q\left(s_{t},a_{t}\right)=\sum_{S_{t+1}\in s_{t}}^{\gamma }p\left(s_{t+1},a_{t}\right)+\gamma^{t}. \end{array}$$

From the above analysis, it is easy to see that rewards are in some sense primary, while the value function as a prediction of rewards is secondary. Without rewards, there is no value, and at the same time, the only purpose of using the value function for prediction is to obtain more rewards. However, the value function is crucial when selecting strategies and evaluating decisions. In an optimization problem, the intelligence makes action choices based on the value function, seeking the action that brings the highest value rather than the highest reward.

## 4. Construction of Tourist Route Identification and Scheduling System

The development of the system is based on six principles: security, comprehensiveness, stability, adaptability, legality, and convenience. The main reasons are the security of the system is fundamental to providing reliable services. First, we must ensure that all users' information is true and reliable, so we must consider how reliable the identity verification is, and all users' information should be well preserved and not leak data. The development of the system must follow six principles, which are security, comprehensiveness, stability, adaptability, legality, and convenience. The comprehensiveness of the system is mainly reflected in two aspects: the first is that the system is designed with full consideration of the entire system operation involved in the institutional sector; at the same time, the second aspect is that the system needs to be continuously maintained and modified in the process of application, so in the process of program design, the use of good comment writing specifications is to ensure a certain space to ensure the expansion of the system [22]. The stability of the system directly determines whether the system is available or not and whether there will be no running errors during the use by users and administrators. The purpose of this system is to provide users with a lot of conveniences and promote certain economic development, while following the relevant regulations of the state in the design process, and must strictly follow the strict national emphasis on information security, which ensures the privacy and security of users. According to the system development principles, the system architecture design and database design are required before the system development.

Mobile travel route recommendation requires obtaining mobile travel-related data from multiple data sources and tracking mobile context and context in real time: first, obtaining user personal information such as name, age, and gender from the registration form; second, obtaining time, geographic location, and location-related context information from the mobile travel platform; and furthermore, obtaining user-attraction association information from the database such as the time of user's choice of attraction. Finally, we extract the existing association rules and classification trees from the external knowledge base as the basis of association rule recommendation. Based on the above important influencing factors, the T-ARC-based mobile travel route recommendation model is established.

The travel route mapped by the income iteration index of the smallest route is the optimal travel route. In this study, the travel recommendation system adopts the current mainstream front-end and back-end separated development model, which can make the front-end and back-end development completely decoupled, the front-end and back-end developers only need to define the interface documents, and then they can synchronize the development without interfering with each other, improving the quality and speed of development [23]. The system uses the Spring Boot framework for back-end development, the Vue framework for front-end development, TensorFlow for model training, and Redis for feature data caching. Based on the functional requirements of the system, this section designs the specific functional modules of the system, which are mainly divided into four parts: home page, attraction recommendation, trip planning, and personal homepage. The specific functions of each part are shown in Figure 2.

Deep learning is based on big data and cannot be separated from the creation of a database after the collection of a large amount of data. The use of artificial intelligence for the development and upgrading of tourism requires the creation of databases for both users and tourism elements. The database for the user is a collection and aggregation of information generated by the user so that the data can be called and processed. In this way, it is possible to gradually add and modify the description and characterization of the selected object over time, and through the collection of data over a long period, it is possible to achieve an exact match with the user's characteristics, so this method is the most common method of database creation. For users, the most important factor at the level of tourism planning is targeted recommendation, and through the establishment of a personal database, the information provided by deep learning also tends to be more personalized and humanized. For tourism resources (such as hotels and attractions), the establishment of a database is a statistical regression on parameters such as the number of user retrievals, hotness, and user feedback, to explore the commonalities and characteristics among attractions [24]. The search for commonality can facilitate the classification of tourism resources, and the search for characteristics can be based on the user database for further recommendations for individuals. Moreover, the feedback on the attention of attractions by the above method can make timely arithmetic processing to predict the crowding level of different attractions. In this process, the crowding level appears as a new parameter to further improve the accuracy of recommendations; at the same time, it can be used as a basis to modify the recommendations for different users, to reasonably allocate and balance the flow of people in scenic spots, avoiding the unbalanced situation of crowding in some scenic spots and scarcity of visitors in others. The establishment of the database is slow to fast and then accurate process, as shown in Figure 3, the system gradually stabilizes after the initial model is established, and the cost of data supplementation and adjustment at a later stage is very low. In summary, the establishment of the personalized database can achieve a fast, accurate, and stable number in tourism design and tourism project recommendation.

Starting from the accommodation center *M*, we visit the seed tourist attractions of the tourist route plan in order and finally return to the accommodation center *M*, forming a closed-loop process, setting the number of tourist attractions visited as *φ*, *φ*=∑_*k*=1_^*m*^*a*_*wk*_. With *M* determined, there are many tourist routes, but not every route maximizes the iterative value of tourist benefits for tourists, and the purpose of this study is to identify the optimal and suboptimal routes for tourists to choose from. The attractiveness and benefit of a certain tourist route to tourists depend on the influence of all factors on that tourist route, including the influence factors *α* and *β* in the actual trip. *α* and *β* are extracted from the Baidu Maps and Gaode Map, and their benefit iteration functions are constructed. The function has the same initial gain iteration value *I*_*O*_ between every two subnodes, i.e., the initialization value *I*_*O*_ is the same when calculating *M* points to other optimal travel seed nodes. Substituting the positive influence factor *α* and the negative influence factor *β* for iteration, the final gain values of the subnodes are output. In a closed-loop structure, the benefit iteration index *L* remains a monotonically increasing function, which increases with the number of visited attractions and finally outputs a maximum value, *L*(*M*, *M*) representing the final return to *M* from the accommodation hotel *M*, completing the whole route tour.

(5) $$\begin{array}{c} L\left(M,M\right)=\sum_{\varphi =1}^{\varphi }h\left(s_{e},s_{e}^{\wedge }\right). \end{array}$$

When 1, compare the sizes of *O*_1_ ≤ *O*_2_, *O*_2_ and *O*_3_; if *O*_2_ > *O*_3_, swap the positions of *O*_2_ and *O*_3_, and then compare the sizes of *O*_2_ and *O*_3_. If *O*_2_ ≤ *O*3, then keep the position unchanged and compare the size of *O*3 and *O*4. Repeat the process until the positions of the elements in the list do not change anymore.

(6) $$\begin{array}{c} x_{0}=E_{u_{i}}^{l}+E_{a_{j}}^{l}. \end{array}$$

After completing the above process, the system outputs an ascending vector *O*_*i*_ of the iterative index of return *L* of a route. According to the above definition, the tour route mapped by the smallest iterative index of the route is the best tour route. Because its output route's gain iteration index sum is the smallest, it means that its gain function value is the largest for all its subnode intervals, representing that tourist can get a better travel experience than other visit orders through the route planning's attraction visit order. In terms of comprehensive output results, the optimal travel route performs best in terms of tourist attraction classification, distance, time, budget expenditure, transportation information service, and tourist attraction star rating. At the same time, the recommendation system also recommends the second-best route and provides visualization of the route for tourists to choose.

## 5. Artificial Intelligence-Aided Image Model Performance Tests

Safety and comfort during travel are also key indicators of comprehensive travel satisfaction. The core of the UPST-TB mobile recommendation algorithm lies in the processing of interest tag sets and the mining of mobile user-interest tag-attraction correlations, and different tag weight preprocessing methods produce different recommendation results, so it is necessary to explore the weighting ratio of the three tag analysis methods in the algorithm. The default rating value of unrated data is 2.5 (on a 5-point scale), the time weight coefficient *ξ* is 0.5, and the minimum similarity between users and attractions *φ* is 0.0001. Calculating the similarity between the user label weight vector ${\overset{⟶}{U}}_{x}$ and the attraction label weight vector ${\overset{⟶}{S}}_{y}$, *U*_*x*_*S*_*y*_ is used to construct a similarity matrix to achieve tourist attraction recommendations. To increase the rationality and interpretability of the algorithm, the experiments were conducted by comparing and analyzing the results of the label weight coefficient *α*, the weighted centrality coefficient *β*, and the label weight diffusion coefficient *γ* at different values and their correlations, and by combining the advantages of the three coefficients, the optimal ratios were determined, as shown in Figure 4.

From Figure 4, the accuracy and recall of the recommendations increase with the increase of *γ* and *β* values and decrease with the decrease of *α* value; the coverage increases with the increase of *α* value and decreases with the decrease of *β*, and *γ* values decrease with the decrease of *β* value, and the change with *β* value is not obvious in the above three figures. It can be determined that the *α* value is positively correlated with the *γ* value and negatively correlated with the *β* value. Therefore, it is not difficult to analyze and obtain that the interesting label weighting coefficients are not highly targeted and have weak performance in accuracy recommendation; the weighted centrality coefficient and label weight diffusion coefficient have better performance in accuracy/recall index, but the recommendation results are too concentrated and inferior to the interesting label weighting coefficients in coverage index, i.e., diversity recommendation. Overall, the evaluation results of all three indicators are better when the value of *γ* is large, and as the coefficient that makes the most use of mobile data, it can be more comprehensive in mining and analyzing user preferences and item attributes. Among them, the weighted centrality coefficient prefers popular tags, the tag weight diffusion coefficient focuses on cold recommendations, the interest tag weight coefficient helps the diversity of recommendations, and the comprehensive performance of the algorithm is improved by combining the three-weight coefficient tuning. Mobile travel recommendation also needs to pay attention to the status of scenic spots, geographical location, situational factors, and contextual information in real time, so as to facilitate tourists to change routes at any time.

The UPST-TB interest label optimization algorithm outperforms both the FolkRank algorithm and UCF algorithm in terms of accuracy and recall metrics for different *n* values and has good performance in accuracy recommendation. Although the accuracy of the UPST-TB algorithm is significantly closer to that of the FolkRank algorithm at *n* = 30, the performance of the UPST-TB algorithm is still clearly superior2. The UCF algorithm based on user preferences is like the FolkRank tag recommendation algorithm in terms of coverage metrics and is always superior, while the UPST-TB algorithm is deficient in diversity recommendation, although it is better at 3. The limitation of collaborative filtering is that it is difficult to handle multidimensional data information, so the UCF algorithm has the worst recommendation effect; the classical FolkRank tag recommendation algorithm is based on the three-part graph and focuses on the correlation between user-tag-item, which is better than the UCF algorithm; the UPST-TB algorithm combines the strengths of both algorithms. Tourists are more inclined to self-planned attractions and routes for flexible self-help travel, tourism application services are gradually transferred to mobile terminals, and smart tourism is deepening and expanding. The UPST-TB algorithm combines the strengths of both algorithms and combines multidimensional data such as user preferences and social tags to make recommendations, which has certain superiority in recommendation performance. Although the label weight diffusion factor is used to mine cold labels and optimize their diversity based on the TF-IDF method, the UPST-TB algorithm still favors popular recommendations and is deficient in diversity recommendations.

To verify the effectiveness of the algorithm, this group of experiments compares the parameter-tuned UPST-TB algorithm with the classical tag recommendation algorithm FolkRank and the user-based collaborative filtering (UCF) algorithm through the core subset of location-set based on tourist attraction recommendations, and the structure is shown in Figure 5.

Experiments prove that the UPST-TB algorithm has advantages in accuracy recommendation, normalizing important mobile information from multiple data sources into interest labels helps improve recommendation performance, and weighting analysis and tuning of the user-interest label set can further optimize the performance of mobile recommendation. The time complexity of the UPST-TB algorithm is O, which is the same as that of the classical algorithm. The UPST-TB algorithm has good performance in the field of mobile travel route recommendation for attraction selection and recommendation. When the number of target points is 10, compared with the d2m-greedy method and the genetic algorithm, the total length of the safe path planned by the MDRP-AC algorithm proposed in this chapter is reduced by 12.00% and 3.11%, respectively.

The runtimes of the graph division for the ParMetis algorithm, GP-Metis algorithm, GraphHash model, and GraphGPU model on each of the three datasets are labeled above the bar graphs. In particular, the runtimes of the exchange optimization phase are marked in square brackets on the bar graphs of the GraphHash and GraphGPU models. The results are shown in Figure 6. The GraphGPU model runs 1.7–2.5 times faster than the ParMetis algorithm and 1.1–1.47 times faster than the GP-Metis algorithm. The algorithms stop the coarsening operation too early in the coarsening phase when dividing large-sized graphs, making the final coarsened graphs too large. In the longitudinal comparison with GraphHash, the GraphGPU optimization phase takes significantly less time than the GraphHash algorithm because the barrel-optimized exchange algorithm in GraphGPU converges in 4–7 iterations, while GraphHash requires 8–13 iterations to converge, which also reflects the effectiveness of the GraphGPU initial clustering division algorithm.

## 6. Simulation Experiment of Travel Route Identification and Scheduling System

The system development process uses the Spring Boot framework for back-end development, Vue framework for front-end, and Python 3.6 language and TensorFlow framework for attraction recommendation service, and the purpose of system functional testing is to detect the operation of each function in the system through test cases. The system is tested and evaluated through the system functional test case table to ensure that the system runs without abnormalities. The test case table contains the case number, name, and prediction result. It mainly tests the functions in the home page, attraction recommendation, itinerary planning, and personal homepage of the travel recommendation system. In the actual multiobjective path planning scenario, the road network information is complex and diverse, and the user needs are different. To make the multiobjective path planning results more suitable for the user's requirements on the safety of travel routes, we use the safety distance between two target points as the distance weight between two target points and verify the effectiveness of the MDRP-AC algorithm proposed in this chapter in the actual. Based on the safe path planning dataset created in Chapter 3 of this thesis, we verify the effectiveness of the proposed MDRP-AC algorithm in urban scenarios. The UPST-TB interest tag optimization algorithm is better than the FolkRank algorithm and the UCF algorithm in terms of precision and recall in different *n* values, and has good performance in accuracy recommendation.

The MDRP-AC algorithm proposed in this chapter models the multiobjective path planning problem as a sequence-to-sequence-based TSP problem constructs an A-Ptr network based on a pointer network specifically designed for solving the TSP problem, and optimizes the parameters of the A-Ptr network by combining the actor-critic algorithm in deep reinforcement learning techniques through the interaction training between the intelligence and the environment to achieve the goal of the shortest total distance of multiobjective point visits. The goal is to predict the output of the sequence and then to achieve the shortest total travel distance of the multiple target points represented by the sequence. The MDRP-AC algorithm, the d2m-greedy method, and the genetic algorithm can obtain good results when the number of target points is 5. As the number of target points increases, the advantage of the MDRP-AC algorithm proposed in this chapter becomes obvious. When the number of target points is 10, compared with the d2m-greedy method and the genetic algorithm, the total length of safe paths planned by the MDRP-AC algorithm in this chapter is reduced by 12.00% and 3.11%; when the number of target points is 20, compared with the d2m-greedy method and the genetic algorithm, the total length of safe paths planned by the MDRP-AC algorithm in this chapter is reduced by 2.98%. The total length of safe paths planned by the MDRP-AC algorithm is reduced by 2.98% and 0.14% compared with the d2m-greedy method and the genetic algorithm, respectively. The results of the safe travel routes corresponding to the three multiobjective point path planning algorithms are shown in Figure 7. From Figure 7, the MDRP-AC algorithm proposed in this chapter effectively reduces the number of users repeatedly passing through the same street in the road network based on the reduction of the total length of the safe path.

From the above experimental results, it can be concluded that the MDRP-AC algorithm proposed in this chapter effectively shortens the total length of multitarget point travel paths, uses the interaction trajectory data obtained from the interaction between the intelligent body and the environment, uses the actor-critic reinforcement learning method to train the pointer network, overcomes the problem of high data cost, reduces the high dependence of network performance on labeled data, and provides a feasible method for multitarget point path planning. Next, we apply the MDRP-AC algorithm to a practical smart travel scenario, design and implement a travel route planning scheme based on the MDRP-AC algorithm, and provide users with personalized path planning recommendations for multiple attractions.

This section designs and implements a travel route planning scheme to be applied to various travel mobile applications. The scheme is based on the MDRP-AC algorithm proposed in this chapter, which uses the shortest distance or safe distance as the distance weight between two target points to achieve the multitarget point access path planning function, i.e., to plan a travel access route based on multiple destinations inputted by the user, and to accomplish the goal of “multisite day trip” travel route planning. Based on the input K destination locations and the user's performance requirements for the path planning results, the distance weights between each two target points are determined by obtaining information about the surrounding streets, intersections, and safety hazard areas from the database. If the user selects the shortest path requirement, task one is executed. The shortest path planning is performed according to the Dijkstra algorithm, and the shortest path planning result of K(K-1)/2 paths is obtained; if the user chooses the safe path demand, task 2 is executed, and the safe path planning is performed according to the Q-SRP algorithm based on the policy guidance mechanism proposed in Chapter 3, 800 iterations of learning are performed according to the starting and ending points of the path, and the safe path planning result of K(K-1)/2 paths is obtained. The path planning result is obtained. The path planning results are stored as sequences in the order of traveling nodes, which can be directly called by the multidestination access path planning task to obtain the distance weights between two destinations. After that, the K destination sequences are input into the AC optimization model containing the A-Ptr network and CL network, 1000 rounds of iterative learning are performed according to the MDRP-AC algorithm process, and finally, the multitarget access sequences are output to obtain the full path planning results, as shown in Figure 8.

We first execute task 2 to get the secure path between every two attractions by Q-SRP algorithm based on the policy-guided mechanism for user B's self-selected multitarget points and the requirement of ensuring path security, use the total length of the secure path as the key index of reward in the MDRP-AC algorithm, and then get the access sequence of these 10 attractions by the MDRP-AC algorithm and the final output of the multitarget point safety path planning results. This scheme can be applied to the path planning of travel mobile applications. According to the user's demand, the planning module can plan the route for users with multiple target points, guarantee the safety and comfort of users in the process of travel, improve user experience, and open a new model of personalized and optimized path planning in smart city and smart tourism scenes.

## 7. Conclusion

This study focuses on the establishment of user-interest sets and deep mining of user-interest tag-item correlation and proposes the UPST-TB mobile recommendation algorithm based on interest tags. By using various data preprocessing methods to weight the interest tags, the quality of tags is further optimized, and the three-part graph data of mobile recommendation are processed in the way of social tag recommendation. An actor-critic-based multitarget point path planning algorithm is proposed. In the multitarget point access sequential path planning task, we want to achieve the optimization objective that multiple target points are all visited once and the total path length is the shortest. Experimental results show that our algorithm results in shorter total path lengths for a larger number of target points compared to distance matrix mapping methods and genetic algorithms used for multiobjective path planning. Finally, the MDRP-AC algorithm is applied to a real travel scenario, and a travel route planning scheme based on the MDRP-AC algorithm is designed and implemented to recommend personalized multispot optimized path planning results for users. In the process of this study, there are still many shortcomings; for example, there are many factors that affect the location recommended routes; in this study, we mainly use user check-in data and attraction review information; in addition to text data, there are weather, time, money, and some other modal data (pictures and audio) that affect the location recommendation, these factors can be incorporated into the model system in future research, and the recommendation mechanism will be more in line with the actual needs.

## Figures and Tables

**Figure 1:** Schematic diagram of stream graph partitioning algorithm classification.

**Figure 2:** System function simple structure diagram.

**Figure 3:** The process of establishing the database of travel route recommendations.

**Figure 4:** Weighting factor test evaluation results.

**Figure 5:** Comparison results of three algorithms.

**Figure 6:** Running time comparison results.

**Figure 7:** Multiobjective point safety path planning results.

**Figure 8:** Full-range path planning results.

## Data Availability

The datasets used and analyzed during the current study are available from the corresponding author upon request.
